# Histopathological Tissue Segmentation of Lung Cancer with Bilinear CNN and Soft Attention

**DOI:** 10.1155/2022/7966553

**Published:** 2022-07-07

**Authors:** Rui Xu, Zhizhen Wang, Zhenbing Liu, Chu Han, Lixu Yan, Huan Lin, Zeyan Xu, Zhengyun Feng, Changhong Liang, Xin Chen, Xipeng Pan, Zaiyi Liu

**Affiliations:** ^1^School of Computer Science and Information Security, Guilin University of Electronic Technology, Guilin, China; ^2^Department of Radiology, Guangdong Provincial People's Hospital, Guangdong Academy of Medical Sciences, Guangzhou, China; ^3^Guangdong Cardiovascular Institute, Guangzhou, China; ^4^Guangdong Provincial Key Laboratory of Artificial Intelligence in Medical Image Analysis and Application, Guangdong Provincial People's Hospital, Guangdong Academy of Medical Sciences, Guangzhou, China; ^5^Department of Pathology, Guangdong Provincial People's Hospital, Guangdong Academy of Medical Sciences, Guangzhou, China; ^6^Department of Radiology, Guangzhou First People's Hospital, The Second Affiliated Hospital of South China University of Technology, Guangzhou, China

## Abstract

Automatic tissue segmentation in whole-slide images (WSIs) is a critical task in hematoxylin and eosin- (H&E-) stained histopathological images for accurate diagnosis and risk stratification of lung cancer. Patch classification and stitching the classification results can fast conduct tissue segmentation of WSIs. However, due to the tumour heterogeneity, large intraclass variability and small interclass variability make the classification task challenging. In this paper, we propose a novel bilinear convolutional neural network- (Bilinear-CNN-) based model with a bilinear convolutional module and a soft attention module to tackle this problem. This method investigates the intraclass semantic correspondence and focuses on the more distinguishable features that make feature output variations relatively large between interclass. The performance of the Bilinear-CNN-based model is compared with other state-of-the-art methods on the histopathological classification dataset, which consists of 107.7 k patches of lung cancer. We further evaluate our proposed algorithm on an additional dataset from colorectal cancer. Extensive experiments show that the performance of our proposed method is superior to that of previous state-of-the-art ones and the interpretability of our proposed method is demonstrated by Grad-CAM.

## 1. Introduction

Lung cancer is the leading cause of cancer-related deaths worldwide [1, 2]. Precise diagnosis is crucial for treatment planning. Histological assessment of hematoxylin and eosin- (H&E-) stained tissue specimens remains the gold standard for lung cancer diagnosis [3, 4]. In clinical practice, pathologists use their domain knowledge and experience to assess the complex morphological and cytological features of tissue samples under a light microscope to diagnose [5, 6]. However, the process is time-consuming, subjective, with considerable inter- and intraobserver variability [3, 7]. Recently, digital pathology, converting conventional glass slides into digital resources known as whole-slide images (WSIs), rises the development of automatic diagnosis [8–10]. One of the most needs for automatic disease diagnosis is to distinguish different tissue components (tumour epithelium, stroma, necrosis, tumour-infiltrating lymphocytes, etc.) in H&E-stained WSIs [11–13]. Therefore, an initial step in automatic diagnosis is to develop a robust automatic tissue segmentation algorithm.

Deep learning models have demonstrated a strong segmentation ability in histopathological images [14–16]. Various DL models have been proposed for patch-level tissue segmentations in WSIs. Xu et al. [15] proposed a DCNN model to extract the convolutional features for classifying epithelial and stromal in histopathological images. Zhao et al. [17] presented a VGG19-based model for automatic tissue segmentation and automated TSR quantification in WSIs of colorectal cancer. Kather et al. [18] compared recently deep learning models in histopathological images in colon cancer and concluded that the VGG19 model worked best at tissue classification. Chan et al. [8] applied a CAM-based method with a fully connected conditional random field for patch-level tissue segmentation. Xu et al. [14] proposed a DenseNet-based approach with focal loss to deal with class imbalance in histopathological images. Anklin et al. [19] proposed a weakly supervised method based on tissue graphs to utilize inexact and incomplete annotations to segment whole-slide images. Yang et al. [20] found that the multimodel method was relatively better than single model-based ones for the automatic diagnosis of lung cancer. Li et al. [21] proposed an EfficientNet-based model to identify tissue in histopathological images. However, they did not take into account the high heterogeneity of tissue types (as shown in Figure 1). Even homogeneous tissue types differ in color, shape, and texture, which provides a further challenge for automatic segmentation.

Bilinear convolutional neural network (Bilinear-CNN) is an effective architecture for fine-grained visual recognition tasks [22–24]. The original bilinear pooling can be generalized to all convolutional neural networks [25]. The bilinear pooling provides an advantage for Bilinear-CNN in that computational layers in networks can have a strong capacity with pairwise interactions [25, 26].

In this paper, we propose a novel Bilinear-CNN-based model to handle the issue of large intraclass variability and small interclass variability in histopathological images. The Bilinear-CNN-based model combines a bilinear convolutional module and soft attention module to perform multitissue classification of histopathological images in lung cancer. It investigates the correct semantic correspondence of intraclass and focuses on the more distinguishable features that make feature output variations relatively large between interclass.

## 2. Materials and Methods

### 2.1. Datasets

In this work, lung cancer and colorectal cancer multitissue histopathological image datasets are used for experiments.

The lung cancer multitissue histopathological image dataset is introduced in this work. It contains 107.7 k patches from 67 slides of lung cancer, which were scanned by an Aperio-AT2 scanner in the Department of Pathology at Guangdong Provincial People's Hospital, China. Each slide corresponds to an independent patient. The training set includes 78 k image patches from 57 slides. The independent test set includes 29.7 k image patches from 10 slides. The image patches are extracted partially overlapping tiles from H&E-WSI images by a sliding window with the resolution of 224 × 224 (20x magnification). The step size of the sliding window is 56 pixels. Within this dataset, tumour epithelium (TUM), stroma (STR), tumour-infiltrating lymphocytes (LYM), necrosis (NEC), bronchus (BRO), vessel (VES), normal (NOR), background (BAC), areas polluted by carbon dust (APC), and others (OTH) can be observed. The dataset is validated by two experienced pathologists and judged by a senior pathologist if there are differences in classification.

The colorectal cancer multitissue histopathological image dataset was published by Zhao et al. [17]. Tissue types were grouped into nine classes, including TUM, STR, LYM, BAC, NOR, debris (DEB), mucus (MUS), smooth muscle (MUC), and adipose (ADP). The training set included 283.1 k image patches from 191 slides. The independent test set included 28.8 k image patches from 48 slides. Then, image patches with the size 224 × 224 (20x magnification) were extracted partially overlapping tiles from H&E-WSI images. The step size of the sliding window was 84 pixels.

### 2.2. Methodology

In this part, we describe our proposed two-stage multitissue segmentation algorithm. First, we introduce a novel Bilinear-CNN-based model to discriminate multiclass tissue types. Second, patches are predicted by our model, then stitched back to get the prediction map. The entire algorithm for automatic tissue segmentation is shown in Figure 2, and an overview of the proposed classification network is shown in Figure 3.

#### 2.2.1. Classification Network

To make feature output variations relatively large between interclass and within the intraclass, we propose a simple but effective method that combined Bilinear-CNN and a soft attention module (Figure 3). The portion of the network to extract the features is ResNet50, because of its outstanding performance in recent computer vision tasks. We remove the global average pooling layer compared to the standard pretrained ResNet50 implementation. Instead, the features extracted by the convolution layer are fed into a bilinear pooling module. Then, a soft attention module is added after the bilinear pooling module and used to receive the features that represented the biological significance of the tissue components, which is the output of the bilinear pooling module. Finally, the softmax layer is used for prediction.

*(1) Bilinear Pooling Module*. The bilinear pooling module [24] is used to investigate the correct semantic correspondence between the intraclass. When given an input feature vector *x* ∈ *R*_*n*_ of a sample, the general linear transformation can be expressed as

(1) $$\begin{array}{c} y=b+w^{T}x, \end{array}$$

where *y* is the output of a node, *b* is the bias, *w* ∈ *R*_*n*_ is the corresponding transformation weight matrix, and the dimension of the input features is *n*.

To investigate the correct semantic correspondence between the intraclass, we use the bilinear pooling module as follows:

(2) $$\begin{array}{c} y=b+w^{T}x+x^{T}F^{T}Fx, \end{array}$$

where *F* ∈ *R*_*k*×*n*_ is the corresponding reciprocity weight matrix with *k* ∈ *N*^+^ factors.

To illustrate the bilinear pool module more clearly, the expression of Equation (2) can be expatiated as

(3) $$\begin{array}{c} y=b+\overset{n}{\underset{i=1}{\sum }}w_{i}x_{i}+\overset{n}{\underset{i=1}{\sum }}\overset{n}{\underset{j=1}{\sum }}\langle f_{i},f_{j}\rangle x_{i}x_{j}. \end{array}$$

The *i*th value of the input *x* is *x*_*i*_. The *i*th variable of the first-order weight is *w*_*i*_, and the *i*th column of *F* is *f*_*i*_. 〈*f*_*i*_, *f*_*j*_〉 is the inner product of *f*_*i*_ and *f*_*j*_, which explains the interaction between the *i*th and *j*th values of the input feature vector.

Compared to other deep learning models, we not only use first-order features but also use second-order features to achieve better classification. The bilinear pooling module can help the convolution layer and full connection layer to break through linear transformation, capture nonlinear features, improve the richness of extracted features, and thus obtain bilinear features of the same subclass, which we use as input into the attention module.

*(2) Soft Attention Module*. The soft attention module [27] receives the bilinear features of the same subclass and increases the feature output variations between different subclass. The attention module provides an attention weight for features that can be participated in backpropagation. First, matrix multiplication between attention weights with feature vector is performed. Then, we get the scalar by using the softmax function, which can be learned with training iterations. Finally, we take the corresponding scalar and matrix multiply each neuron, and sum to get the distinguishable features as follows:

(4) $$\begin{array}{c} c=\overset{n}{\underset{i=1}{\sum }}a_{i}f_{i}, \end{array}$$

where *c* is the distinguishable feature, *a*_*i*_ is the *i*th variable of the attention weight *a*, and *f*_*i*_ is the *i*th value of the input feature *y* from Equation (3).

The expression of the differentiable *a* can be explained as

(5) $$\begin{array}{c} a_{i}=\frac{\exp\left(e_{i}\right)}{\sum_{i=1}^{n}\exp\left(e_{i}\right)}, \end{array}$$

where *e*_*i*_ is *i*th value of the scalar and *e* is expatiated as

(6) $$\begin{array}{c} e=\overset{n}{\underset{i=1}{\sum }}w_{i}f_{i}, \end{array}$$

where *w*_*i*_ is *i*th variable of the attention weight, which can be learned with training iterations.

The soft attention module can improve the ability of the model to learn distinguishable features of different subclass in histopathological images. The scalar is used to make the model focus on the more distinguishable features, and with the learning, important distinguishable features become more prominent in the model. And we have demonstrated the effectiveness of this method through experiments. The details of the experiments are shown in Section 2.3.

#### 2.2.2. Transfer Learning

In the lung multitissue histopathological image classification task, the classification network pretrained with transfer learning. This strategy can make better use of existing public multitissue histopathological image datasets and achieve better results on the multitissue classification task. We used the Bilinear-CNN-based model trained on colorectal cancer multitissue histopathological image dataset as the pretrained model. And then, we fine-tuned the model in the lung multitissue histopathological images dataset based on the pretrained model.

#### 2.2.3. Visual Interpretability of the Classification Network

To demonstrate that the Bilinear-CNN-based model can identify the tissue types, we utilized the Grad-CAM to generate the visual interpretability of the classification network. Grad-CAM [28] describes a visual explanation of models based on object gradients. A localization map of important image regions is highlighted by Grad-CAM. In the decision-making process, the gradient information flowing into the last convolutional layer of the CNN is utilized by Grad-CAM to assess the importance of features.

#### 2.2.4. Segmentation Map

The trained Bilinear-CNN-based model is used for patch-level multitissue segmentation on histopathological images, and a predictive segmentation map is generated. The detailed operations are as follows. First, we use OpenSlide software to downsample the WSI of lung cancer to get the tissue mask. To distinguish tissue from the background, the tissue region is obtained by threshold segmentation algorithm from the tissue mask. Overlapping tiles are extracted partially by a sliding window with a size of 224 × 224 from the tissue region. The step size of the sliding window is set at 128 pixels. Then, each image tile is input into the trained multitissue classification model to generate a prediction probability. Finally, the tissue class with the highest prediction probability is selected as the classification result of the image tile.

### 2.3. Implementation and Training Details

The study was implemented with the open-source software library PyTorch version 1.6.0 on a workstation with Intel(R) Core(TM) i5-10600KF CPU, 32 GB memory, and equipped with NVIDIA GeForce 3090 GPU. During training, the augmentation techniques were applied for the training dataset, including rotations, normalized color appearance, and horizontal flipping. All models in this implementation received input patches of size 224 × 224. All models were trained with a batch size of 32, weight decay of 1*e* − 4, and momentum of 0.9 for 80 epochs. Adam optimization with a learning rate of 3*e* − 4 was used on the colorectal cancer multitissue histopathological image dataset. We used Adam optimization with an initial learning rate of 3*e* − 4, and then, it reduced to one-tenth if the loss stopped reducing for 30 epochs on the lung cancer multitissue histopathological image dataset.

## 3. Results

We made independent comparisons to the evaluated model on the lung cancer dataset and an additional dataset from colorectal cancer. Our proposed model was compared to state-of-the-art approaches recently used in computer vision and models specifically designed for the task of tissue classification.

### 3.1. Comparison on the Lung Cancer Dataset

For comparison of existing models on the lung cancer dataset, all models were pretrained on the colorectal cancer dataset. The results of the comparison are shown in Tables 1 and 2.  Figure 4(a) shows the comparison between the ResNet50 model with a bilinear pooling module and attention module and other models concerning the loss on the lung cancer dataset. The loss of the proposed model decreases much faster and smoother than that of other models, demonstrating its superior convergence speed. The ResNet50 model with bilinear pooling module and attention module achieves the best performance.

To analyze which image regions the proposed model focused on, heatmaps of different models are shown in Figure 5. A localization map of important image regions in heatmaps is highlighted by Grad-CAM. Heatmaps of the four most common tissue types are shown, and the slides of lung cancer scanned in 20x magnification factor are selected at random. Figure 5 shows the heatmaps of different models by Grad-CAM which highlights the importance of regions for classification and demonstrates a better focus of the ResNet50 model with bilinear pooling module and attention module on histopathological regions than classic CNNs.

### 3.2. Comparison on the Colorectal Cancer Dataset

To further evaluate our proposed algorithm, the comparative experiments on an additional dataset from colorectal cancer were implemented. On the colorectal cancer dataset, the pretrained model with ImageNet was used. ImageNet is a large image dataset containing hundreds and thousands of images. In transfer learning tasks, ImageNet is usually used for pretrained models. This public dataset was used to assess the generalization ability and robustness of our multitissue classification model. The results of the comparison are shown in Tables 3 and 4.  Figure 4(b) shows the comparison between the ResNet50 model with a bilinear pooling module and attention module and other models concerning the loss on the colorectal cancer dataset. The loss of the proposed model converges faster than in other models. The results illustrate that the proposed model combines the bilinear pooling module and soft attention module to make feature output variations relatively large between interclass and within the intraclass, learn the distinguishable features, and improve the accuracy of the multitissue classification task.

Several conclusions can be drawn: (1) The result of the proposed method is superior to state-of-the-arts recently. (2) the ResNet50 model with bilinear pooling module and attention module achieves the highest classification accuracy in the test, and it is shown that the Bilinear-CNN-based model works well on the multitissue task and effectively alleviates the problem of large intraclass variability and small interclass variability. (3) The model combined Bilinear-CNN, and soft attention module is suitable for the multitissue task.

### 3.3. Visualizing the Segmentation Results of WSIs

The segmentation result of H&E-stained WSIs in lung cancer is drawn as a map covered on the tiles with various colours representing the output tissue types. In Figure 6, colour standing for each tissue type is randomly selected. The predictions of tissue types are observed and mapped to the in situ tissues. Our method obtains the tissue mask of the downscaled WSI. A threshold segmentation algorithm is used to distinguish tissue from the background and then get the tissue region from the tissue mask. Figure 6 also shows that the predicted regions by our classifier are highly consistent with the distribution of tissue types in histopathological images.

## 4. Discussion

Automatic tissue segmentation is faced with a challenge in that whole-slide images usually have a large resolution and cannot be directly fed into CNNs. This challenge cannot be alleviated by resizing the image size, which causes the loss of much information. Moreover, in the study of lung cancer histopathological images, the existing works are basically based on the backbone of natural image classification to identify the tissue types. In addition, compared with natural images, histopathological images are high heterogeneity in different tissue types with large intraclass variability and small interclass variability.

To address these issues, we propose a two-stage automated tissue segmentation framework. In the first stage, large resolution WSIs are cut into small patches and then feed into the proposed classification model to predict separately. To alleviate the issue of large intraclass variability and small interclass variability, we introduce a Bilinear-CNN-based classification model. In previous studies, Kather et al. [18] used the VGG model to extract deep learning feature to identify tissue types. In Results, experimental results show that the VGG model does not perform well in the face of high heterogeneity of multiple tissue types. It is guessed that the model is designed for natural images and does not take into account the subtle features of pathological images. Chan et al. [8] improved the CNN model combined with Grad-CAM for the segmentation and classification of histological images. It relies on the task-specific postprocessing steps and generalizes poorly. Different from the previous approaches, this Bilinear-CNN-based classification network investigates the correct semantic correspondence between the intraclass by bilinear convolutional module and focuses on the distinguishable features of the interclass by soft attention module. The classification network can capture subtle features of pathological images well. The classification result of the proposed method is superior to state-of-the-arts recently. In addition, Figure 4 shows the proposed model has the fastest convergence speed than that of other models. Heatmaps generated by Grad-CAM provide visual interpretability of the classification results. It shows that this network is more sensitive to histopathological regions than classic CNNs. In the second stage, the classification results are stitched tile by tile to implement automatic tissue segmentation. Zhao et al. [17] input each image tile of entire WSI into the CNN model, including the background. In our method, the threshold segmentation algorithm is introduced to distinguish the tissue region from the background, and then, the category prediction of the tissue region is carried out. Compared with directly traversing the whole WSI, a large number of redundant computing overhead is reduced and the efficiency of WSI segmentation is improved.

Although our method is effective for lung cancer segmentation, some limitations remain. Our method uses the histopathological dataset for pretrained models to accelerate the training convergence. However, the histopathological dataset is not as convenient as ImageNet for different models because there are no prepared pretrained models like ImageNet. Moreover, the result of segmentation is patch-level, which is roughly compared with semantic segmentation. But the proposed framework uses image-level annotations to complete the segmentation tasks. Image-level annotations are easier to obtain than pixel-level annotations. Therefore, bridging the gap between image-level annotations and pixel-level segmentation will be the focus of the future investigation.

## 5. Conclusions

In this paper, we propose an automated tissue segmentation framework with two stages. In the first stage, the classification model combines a bilinear convolutional module and soft attention module to improve the accuracy of tissue classification. In the second stage, the threshold segmentation algorithm distinguishes tissue from the background to avoid redundant computing of the background. The framework completes the tissue segmentation task via utilizing the image-level annotations.

## Figures and Tables

**Figure 1:** Example images of the (a–d) tumour epithelium and (e) stroma. Tumour epithelium (a–d) has large intraclass variability. (e) Stroma has small interclass variability with (c) tumour epithelium.

**Figure 2:** An overview of the proposed multitissue segmentation algorithm. Stage 1: a classification network is pretrained on the colorectal cancer dataset, and transfer learning is used to train the classification network with the training set of the lung cancer dataset. The independent image dataset is used to evaluate the classification accuracy of the network. Stage 2: H&E-WSI image (20x magnification) is segmented through stitching the classification results tile by tile. H&E: hematoxylin and eosin; WSI: whole-slide image; TUM: tumour epithelium; LYM: tumour-infiltrating lymphocytes; STR: stroma; NOR: normal; VES: vessel; BRO: bronchus; NEC: necrosis; APC: areas polluted by carbon dust; BAC: background; OTH: others.

**Figure 3:** An overview of the proposed classification network. First, the images are fed into ResNet50 to get the feature maps, and feature maps are input to the bilinear function to obtain the bilinear vector; then, the attention weight is got from the attention function, and finally, the bilinear vector multiplies the attention weight to obtain the attention feature flowed into the softmax layer for classification.

**Figure 4:** Convergence analysis of models. Implementation and training details of all models are consistent with Section 2.3. (a) Loss on lung cancer dataset. (b) Loss on colorectal cancer dataset. (1) EfficientNet, (2) DeepTissue Net, (3) VGG19, (4) ResNet50, and (5) ResNet50 model with bilinear pooling module and attention module.

**Figure 5:** Heatmap of different models generated by Grad-CAM. (a) Slides of lung cancer scanned in 20x magnification factor, (b) heatmap of DeepTissue Net, (c) heatmap of ResNet50, (d) heatmap of the ResNet50 model with bilinear pooling module and attention module. It shows that the ResNet50 model with bilinear pooling module and attention module can detect the largest histopathological region. TUM: tumour epithelium; STR: stroma; LYM: tumour-infiltrating lymphocytes; NEC: necrosis.

**Figure 6:** (a) Examples of H&E-stained WSIs in lung cancer and (b) corresponding segmented results.

**Table 1:** Results on lung cancer dataset (all models pretrained on colorectal cancer dataset).

Model	Average precision	Average recall	Average F1
ResNet50 [29]	0.9239	0.9279	0.9259
VGG19 [30]	0.9185	0.9238	0.9211
EfficientNet [31]	0.9184	0.9295	0.9239
DeepTissue Net [14]	0.9218	0.9250	0.9234
ResNet50+bilinear pooling module	0.9253	0.9286	0.9269
ResNet50+attention module	0.9268	0.9291	0.9279
ResNet50+bilinear pooling module+attention module	0.9394	0.9415	0.9404

**Table 2:** The classification F1 score of tissue types on lung cancer dataset.

Model	TUM	LYM	STR	NOR	VES	BRO	NEC	APC	BAC	OTH
ResNet50 [29]	0.9686	0.9914	0.8687	0.8532	0.8512	0.9615	0.9668	0.9962	0.9959	0.7734
VGG19 [30]	0.9639	0.9913	0.8720	0.8354	0.8821	0.9545	0.9628	0.9939	0.9944	0.7219
EfficientNet [31]	0.9514	0.9789	0.8854	0.8414	0.8768	0.9533	0.9689	0.9955	0.9957	0.7326
DeepTissue Net [14]	0.9331	0.9640	0.8669	0.8635	0.8973	0.9542	0.9589	0.9967	0.9915	0.7852
ResNet50+bilinear pooling module	0.9698	0.9911	0.8753	0.8658	0.8736	0.9538	0.9638	0.9969	0.9936	0.7857
ResNet50+attention module	0.9712	0.9916	0.8862	0.8732	0.8954	0.9582	0.9615	0.9972	0.9931	0.7516
ResNet50+bilinear pooling module+attention module	0.9739	0.9911	0.9056	0.8788	0.9186	0.9586	0.9766	0.9952	0.9935	0.8025

**Table 3:** Results on colorectal cancer dataset (all models were pretrained on ImageNet).

Model	Average precision	Average recall	Average F1
VGG19 [30]	0.9650	0.9660	0.9655
DeepTissue Net [14]	0.9770	0.9775	0.9772
EfficientNet [31]	0.9779	0.9784	0.9781
ResNet50 [29]	0.9736	0.9746	0.9741
ResNet50+bilinear pooling module	0.9764	0.9771	0.9767
ResNet50+attention module	0.9789	0.9794	0.9791
ResNet50+bilinear pooling module+attention module	0.9823	0.9826	0.9824

**Table 4:** The classification F1 score of tissue types on colorectal cancer dataset.

Model	TUM	STR	LYM	MUC	MUS	NOR	BAC	DEB	ADI
VGG19 [30]	0.9870	0.9266	0.9773	0.9748	0.9662	0.9720	0.9586	0.9642	0.9580
DeepTissue Net [14]	0.9806	0.9413	0.9722	0.9784	0.9742	0.9806	0.9988	0.9711	0.9958
EfficientNet [31]	0.9814	0.9569	0.9827	0.9665	0.9671	0.9818	0.9982	0.9718	0.9942
ResNet50 [29]	0.9756	0.9243	0.9673	0.9852	0.9568	0.9866	0.9978	0.9729	0.9972
ResNet50+bilinear pooling module	0.9787	0.9502	0.9808	0.9614	0.9602	0.9869	0.9978	0.9771	0.9940
ResNet50+attention module	0.9803	0.9554	0.9810	0.9667	0.9826	0.9851	0.9974	0.9673	0.9940
ResNet50+bilinear pooling module+attention module	0.9860	0.9591	0.9845	0.9763	0.9693	0.9879	0.9982	0.9830	0.9966

## Data Availability

Previously reported colorectal cancer data was used to support this study and is available at doi:10.5281/zenodo.4024676. This prior study (and dataset) is cited at a relevant place within the text as Reference [17]. The lung cancer data used to support the findings of this study have not been made available because of third-party rights. The code will be available at https://github.com/Hellowmyname/bcnn_attention_lung.
